The article "The Application of Ultrasound Image in Cancer Diagnosis" was retracted in 2023. Reasons: signs of a paper mill; compromised peer review; unreliable results or conclusions.

# The Application of Ultrasound Image in Cancer Diagnosis

**DOI:** 10.1155/2021/8619251

**Published:** 2021-11-09

**Authors:** Xiaoli Wang, Mei Yang

**Affiliations:** Department of Ultrasound, Gansu Provincial Hospital, Lanzhou 730000, Gansu, China

## Abstract

In order to solve the problem of low accuracy, high cost, and difficult detection of traditional algorithms, a new algorithm based on ultrasound imaging is proposed in this paper. The algorithm is based on fuzzy clustering to diagnose the disease and effectively improve the accuracy of the algorithm. By testing the actual scene, it effectively proves the effectiveness and accuracy of the algorithm, which can find and treat diseases in time and can be widely used and popularized in clinical research in China.

## 1. Introduction

With the development of society, in recent years, the incidence of breast diseases in my country has been increasing, among which malignant breast tumors are more serious [1, 2]. This disease has a major impact on women's health and gradually develops towards younger age [3, 4]. This study will use the comparative method to compare clinical case diagnosis and ultrasound imaging [5, 6]. Breast disease is a disease originating from breast glands, fat, lymph, blood vessels, nipples, and other breast-related tissues. Breast diseases include inflammatory diseases, benign breast lesions, malignant breast tumors, congenital abnormalities, and male breast development.

In view of the application research of ultrasound imaging in cancer diagnosis, some researchers conducted research on the diagnosis of lung cancer by fine-needle aspiration biopsy guided by bronchial ultrasound. 73 patients with suspected lung cancer who were examined by EBUS-TBNA from 2013 to 2015 were selected for the fine-needle aspiration biopsy, and then analysis of the results showed that the positive rate of EBUS-TBNA lung biopsy was 76.8%, so it is feasible to use ultrasound-guided fine-needle aspiration biopsy to diagnose lung cancer [7]. Some researchers have studied the pathological state of the axillary lymph node (ALN) and proposed that ALN plays a vital role in the diagnosis and treatment of breast cancer patients. Therefore, they proposed the use of real-time elastography (RTE) and grayscale ultrasound to generate a scoring system. It is used to evaluate the pathology and breast cancer status of patients with axillary lymph nodes (ALN) and verify it through experimental methods. 97 people with breast cancer were selected, and pathology for patients with axillary lymph nodes (ALN) was performed. With the assessment of breast cancer status, the experimental results showed that the scoring system is actually effective [8]. In addition, some researchers have conducted research on the application of ultrasound in the diagnosis of cervical cancer and selected 61 patients with cervical cancer confirmed by surgical pathology before surgery and MRI and other data to review them. The main purpose is to detect ultrasound. The accuracy rate and the influence of MRI were analyzed. The experimental results showed that 57 cases of ultrasound showed abnormalities, the uterus was irregularly enlarged, the shape of the cervix was abnormal, and the echo would make the diagnosis of unbalanced changes in MRI effective [9]. Some researchers have conducted research on the application of tumor abnormal protein (TAP) combined with ultrasound in the diagnosis of early endometrial cancer. 248 patients with suspected endometrial cancer in the women's hospital from 2013 to 2015 were selected and divided into two groups: one is the control group and the other is the observation group. The control group is subjected to routine ultrasound examination, and the observation group is combined with tumor abnormal protein (TAP) for examination. By comparing the differences in the diagnosis results of the two methods, the overall diagnostic coincidence rate for endometrial lesions by routine ultrasound examination was 87.90%, and the diagnosis coincidence rate for early endometrial cancer combined with tumor abnormal protein examination was 94.67% (*n* = 71). It can be seen that the combined tumor accuracy of abnormal protein detection is higher, so the method of tumor abnormal protein (TAP) combined with ultrasound examination is worthy of promotion in clinical practice [10]. In summary, there are still many research results on the application of ultrasound in cancer diagnosis, and there are few researches on the feature analysis of ultrasound images. Characteristics of ultrasound diagnostics are as follows: ultrasound has good resolution to human soft tissue and is conducive to identifying small lesions of biological tissue. The ultrasound image shows that the required image can be obtained without staining, which is conducive to the detection of living tissue. There are many methods to display ultrasonic information, such as A-mode, B-mode, M-mode, C-mode, and Doppler ultrasound. It can be used according to different needs to obtain variety of information and achieve the effect of wide application.

This paper focuses on the application of ultrasound imaging in cancer diagnosis, makes a general summary of the application of ultrasound imaging in cancer diagnosis on the basis of relevant literature data, and then conducts experimental research on the application of ultrasound imaging in breast cancer diagnosis. Mainly by analyzing the ultrasound images of the patients again, the accuracy of diagnosis is analyzed first, then the features of the ultrasound images are summarized, and the application value of ultrasound images in the diagnosis of breast cancer is obtained from the results. Note that ultrasonic image reflects the difference of acoustic parameters in the medium and can obtain information different from optics, X-ray, y-ray, and so on. Ultrasound has good resolution to human soft tissue and can obtain useful signals with a dynamic range of more than 120 dB, which is conducive to the identification of small lesions in biological tissue. When ultrasound images show living tissues, the required images can be obtained without staining.

## 2. Ultrasound Imaging Research

### 2.1. Application of Ultrasound Imaging in Cancer Diagnosis

1. Morphological diagnosis of visceral lesions and general anatomical examination of organs: ultrasonic diagnosis can perform tomographic images of various organs according to the changes in tissues and the morphological changes of pathological anatomy related to the image. The image and morphological manifestations are consistent, and localization and qualitative diagnosis can be achieved based on tomographic image lesions [11].
2. Functional study of changes in ultrasound images or Doppler ultrasound spectrum produced by the physiological characteristics of certain organs and tissues: echocardiography and Doppler ultrasound can be used to detect double power systolic and diastolic function, blood flow and blood flow measurement, gallbladder swelling and gastric function discharge, respiratory diaphragm activity, and so on [12]. Doppler ultrasound can be divided into pulse Doppler, continuous Doppler, high pulse repetition rate Doppler, multipoint gated Doppler, and color Doppler flow imaging. In the case of two-dimensional echocardiography positioning, it uses the Doppler principle and a series of electronic technologies to display the spectrum of blood flow of a certain volume (SV) at a certain point in the heart or large blood vessels in real time. It is a noninvasive technique for detecting intracardiac shunt and reflux [13–15].
3. Through ultrasound infiltration experiments, invasive ultrasound not only closely combines ultrasound diagnosis with clinical pathological cytology, biological systems, and other technologies but also improves the diagnostic capabilities of ultrasound. It can also be used to guide ultrasound needle puncture and inject therapeutic drugs or use laser, microwave, and other means to remove effusion, bleeding, and abscess, thereby increasing the clinical application of ultrasound. The enhancement effect of ultrasound can be as a result of thermal, mechanical, and chemical changes of biological tissues caused by ultrasound. The thermal effect is the result of absorbing the ultrasonic mechanical force of the medium and interface, and the mechanical energy of the sound field is constantly transformed into heat. Ultrasound can cause deep penetration temperature, which may increase the diffusion and solubility of penetrant and may also lead to vasodilation and increase blood flow, making skin vascular penetration easy to occur.

### 2.2. Ultrasound Image-Related Formula

Ultrasound images are mainly affected by multiple factors such as sound wave frequency, blood flow velocity, and the relative angle between the sound beam and the blood flow direction. The relationship between them is shown in the following Doppler equation:

(1) $$\begin{array}{c} \text{Df}=\frac{2fv\;\cos\;\theta }{c}, \end{array}$$

where Df = Doppler shift frequency (the difference between the transmit frequency and the receive frequency), *f* = transmit frequency, *v* = blood flow velocity, *θ* = angle between sound beam and blood flow, and *c* = sound wave velocity (1540 m/s).

Note that when two or more sound waves meet, they will add or subtract from each other and influence and stack each other. This phenomenon is called wave interference. If their peaks and troughs are completely in phase, they strengthen each other, so the amplitude of the resulting waveform is higher than that of any single waveform. If the peaks and troughs of the two waveforms are completely out of phase, they will cancel each other, resulting in no waveform at all.

### 2.3. Segmentation Algorithm of Ultrasound Images

The FCM algorithm only uses pixel gray information and does not consider pixel space information. For very noisy images, this may result in incorrect pixel classification. Ultrasound images contain a lot of noise. To improve the FCM algorithm, the influence of grouping noise must be considered. The method is as follows.

First, define a spatial function:

(2) $$\begin{array}{c} h=\sum_{k\in \text{NB}\left(x\right)}\mu_{ik}. \end{array}$$

NB (*x*) represents a square window centered on pixel *x* and *h* represents the degree to which the pixel *x* belongs to the *i*-th category. The meaning of *h* is that if its neighborhood is more likely to belong to a certain category, then the pixel is more likely to belong to this category. The new iterative formula obtained from this is

(3) $$\begin{array}{c} \mu =\frac{\mu^{p}h^{q}}{\sum_{k=1}\mu_{kj}^{p}h_{kj}^{p}}, \end{array}$$

where *p* and *q* control the proportion of *u* and *h*. For uniform images, the introduction of *h* will not change the clustering results. For noisy images, the introduction of neighborhood information reduces the impact of noise. In this way, the misclassification caused by noise will be corrected.

In addition, using the characteristics of unsupervised fuzzy clustering calibration of fuzzy C-means (FCM) for image segmentation can reduce human intervention and is more suitable for the characteristics of uncertainty and fuzziness in the image. FCM algorithm is very sensitive to initial parameters. Sometimes it needs manual intervention in parameter initialization to approach the global optimal solution and improve the segmentation speed. In addition, the traditional FCM algorithm does not consider spatial information and is sensitive to noise and uneven gray level.

## 3. Application Experiment of Ultrasound Imaging in the Diagnosis of Breast Cancer

### 3.1. Experimental Design Analysis

In this paper, the application of ultrasound imaging in breast cancer diagnosis is experimentation. Therefore, targeted breast cancer patients are selected for experimental research. By analyzing the breast ultrasound images of patients, we summarize some relevant laws and provide some basis for breast cancer diagnosis.

### 3.2. Data Sources

The experimental patients came from breast cancer patients in the gynecology hospital of the city. First of all, the willingness of the patients in the hospital was investigated. A total of 74 patients were tested. The total number of patients willing to do the experiment was 67, and the main age was 19–79 years.

### 3.3. Analysis of Ultrasound Diagnosis of Breast Cancer

(1) The shape is irregular with an uneven surface. (2) The internal echo is very low, the necrosis caused by heavy bleeding is irregular, and there is no echo. (3) There are edge changes such as “abrasion” or “malignant halo” on the edge of the mass. (4) The echo at the rear gradually attenuates. (5) The size ratio is >1. (6) Small calcifications may occur inside the mass, distributed in groups. (7) The mass and surrounding tissues are compressed, and the cooper ligament increases thickness. Based on a two-dimensional grayscale image, a color Doppler function is used.

It is consistent with the classification according to the semiquantitative analysis of blood flow: (1) Grade 0, no large blood flow occurred and no obvious mass. (2) Grade II: the mass has 3 to 4 blood flow points or large primary blood vessels; there are many small blood vessels. (3) Grade II: there is a lot of blood flow, and more than 4 blood vessels are visible. 0 to I are benign masses, and II to II are breast cancers. Based on color Doppler, by using Doppler spectrum technology to measure peak systolic flow velocity and vascular resistance index, PSV > 20 cm/st10 and RI > 0.71l1 are diagnosed as breast cancer.

By observing whether there are localized lesions in the breast gland, the shape, boundary, internal echo, blood flow distribution, and spectrum characteristics can effectively judge the nature of the lesions. For the mass found by palpation and the mass or dense small calcification found by breast X-ray examination, we should carefully check whether there are localized lesions.

### 3.4. Choice of the Instrument

The test equipment is Acuson Sequoia 512, a color ultrasound instrument launched by Siemens in Germany. The sensor model and measuring frequency are 6C2-S, 4.0～6.0 MHz.

The contrast agent, SonoVue, is a microbubble ultrasound agent whose main component is the inert gas sulfur hexafluoride (SF6), and its surface is coated with a layer of phospholipid to maintain the strength of the microbubbles. The specification formulated by Bracco (Italy) is a 60 mg dry powder formula. Before use, dissolve 60 mg of SF6 dry powder preparation in 6 ml of normal saline and shake well for later use. During the angiography, 2.5 ml of intravenous suspension was drawn for rapid bolus injection, followed by rapid injection of 4.0 ml of normal saline into the tube. Once the microbubbles enter the blood vessel, they amplify the signal-to-noise ratio of the image by amplifying the harmonic signals of the blood. The diameter of the microbubbles is about 3 to 5 *μ*m, and the patient can remove them from the body through a breathing cycle of about 20 minutes.

### 3.5. Ultrasonic Inspection Methods

In the field of image processing, region of interest (ROI) is an image region selected from an image, which is the focus of image analysis. Delineate the area for further processing. Using ROI to circle the target you want to read can reduce processing time and increase accuracy. In order to facilitate postdifferentiation analysis, including the transfer of the entire wound and part of the normal gland tissue to contrast conditions, the process is displayed in double frames in real time; that is, two-dimensional images, grayscale images, and ultrasound images on the same plane are displayed at the same time. After appropriately adjusting the grayscale, depth, and focus according to the size and position of the tumor, the prepared contrast agent (SonoVue) is quickly injected through the cubital vein, and then 5 ml of normal saline is quickly injected. The dynamic data storage button and the screening time are activated at the same time during the examination, instructing the patient to continue breathing calmly. Try to determine the position and angle of the catheter to ensure that the return on investment during the entire imaging process remains the same. The storage time is 180 s. During the imaging process, observe the image of the wound. If necessary, it can be observed for up to 8 minutes. After angiography, if there is no discomfort, the patient will stay for 25 minutes and then leave.

### 3.6. Observation Indicators

Judge the accuracy of the patient's diagnosis. In the benign group, the patient was found to have a small obvious lump or thick skin, and the patient's nipples were sunken to prevent axillary lymph node metastasis. The tumor in the malignant group was crab-shaped, with no internal capsule, subsonic velocity, uneven distribution of dark areas, spots, no echo or subsonic velocity, multivessels, and high-frequency impedance.

### 3.7. Statistics

SPSS is the earliest statistical software in the world that uses a graphical menu-driven interface. Its most prominent feature is that the operation interface is very friendly, and the output results are beautiful. It shows that almost all functions in a unified and standardized interface use the windows window to show the functions of various data management and analysis methods, and the dialog box shows various function options. As long as users master certain windows operation skills and master the principle of statistical analysis, they can use the software to serve specific scientific research work. In addition, the analysis results are clear, intuitive, and easy to learn and use and can directly read excel and DBF data files. It has been extended to computers with various operating systems. It, together with SAS and BMDP, is known as the three most influential pieces of statistical software in the world.

We used Excel 2010 to establish a database and we used SPSS 20.0 to perform statistical analysis on the data, with perforation or surgical pathological results as the gold standard. The calculated data is represented by (*x* ± *s*), the comparison between the two groups uses the classification test of two independent samples, and the calculated data uses the *t*-test to calculate the sensitivity, specificity, and accuracy of breast cancer. *P* < 0.05 indicates that there is no statistical significance of variability.

## 4. Analysis of Experimental Results

### 4.1. Analysis of Basic Patient Data

The analysis of some basic data of the patients in this article can exclude the influence of other factors on the experiment. The basic data of the patients are shown in Table 1.

It can be seen from Figure 1 that breast cancer patients are mainly between 20 and 40 years old. This is mainly because women are under greater pressure at this stage and they do not pay too much attention to physical examinations, and most of the patients are benign. Malignant breast cancer mainly occurs between the ages of 40 and 60. At this stage, the physical fitness of women begins to decline, and women are facing menopause.

### 4.2. Comparison of the Characteristics of the Sound Image after Radiography

A comparative analysis of the characteristics of the sound image after the radiography and the relevant data results are shown in Table 2.

It can be seen from Figure 2 that the main features of the ultrasound image after contrast enhancement are 20/29 for high enhancement and 19/29 for uneven enhancement. After enhancement, the boundary of the mass is not clear 18/34 and penetration, twisting of blood vessels, or blood vessels can be seen around the mass radial enhancement; then, there is no irrigation area in the lesion.

### 4.3. Analysis of the Accuracy of Ultrasound Images

The accuracy analysis of ultrasound images is to compare the ultrasound diagnosis of several breast cancer types with the actual results. The relevant data results are shown in Table 3.

It can be seen from Figure 3 that the accuracy of the diagnosis of breast cancer using ultrasound imaging is still relatively high, the accuracy rate is above 98%, and the number of errors is very small.

### 4.4. Comprehensive Scoring Results of Contrast-Enhanced Ultrasound

According to the comprehensive score of the contrast-enhanced ultrasound results, grades 1–3 are benign and 4-5 are malignant. The relevant data results are shown in Table 4.

It can be seen from Figure 4 that a total of 26 breast masses were rated as benign and 40 breast masses were rated as malignant. From this, it can be seen that the diagnostic accuracy of ultrasound imaging is still relatively high.

## 5. Conclusions

Aiming at the problems of low efficiency, low precision, and long time-consuming in the process of tumor diagnosis and detection, the existing traditional algorithms are difficult to judge accurately. This paper can accurately identify and detect relevant tumors by using the strategies of fuzzy clustering and image processing and effectively replace the traditional human resources. A large number of experiments show the effectiveness and superiority of this algorithm; thus, we can effectively avoid mass metastasis.

## Figures and Tables

**Figure 1:** Analysis of basic patient data.

**Figure 2:** Comparison of the characteristics of the sound image after radiography.

**Figure 3:** Analysis of the accuracy of ultrasound images.

**Figure 4:** Comprehensive contrast-enhanced ultrasound score.

**Table 1:** Analysis of basic patient data.

	Benign	Malignant
20–40	20	10
40–60	5	25
60–80	4	3

**Table 2:** Comparison of the characteristics of the sound image after radiography.

	Benign	Malignant
Strength	18	13
	11	25

Enhancement direction	20	20
	9	18

Contrast agent distribution form	19	18
	10	20

Border after angiography	18	14
	11	24

Peripheral penetration or radial enhancement	22	13
	7	25

Internal perfusion defect	21	15
	8	23

**Table 3:** Analysis of the accuracy of ultrasound images.

	Ultrasound imaging diagnosis	Clinicopathological diagnosis
Benign mass	12	13
Purulent breast mass	10	11
Breast cyst	9	10
Breast fibroma	8	8
Breast lobular hyperplasia	7	7
Malignant mass	6	7
Invasive ductal carcinoma of the breast	5	5
Ductal papillary carcinoma of the breast	5	5
Medullary breast cancer	4	4
Malignant cystosarcoma phyllodes of the breast	2	2

**Table 4:** Comprehensive contrast-enhanced ultrasound score.

	Benign	Malignant
1	3	2
2	6	2
3	10	3
4	18	4
5	2	18

## Data Availability

The data underlying the results presented in the study are included within the manuscript.
